The article "Simulation of Automatic Color Adjustment of Landscape Image Based on Color Mapping Algorithm" was published in 2022. Journal: Comput Intell Neurosci.

# Simulation of Automatic Color Adjustment of Landscape Image Based on Color Mapping Algorithm

**DOI:** 10.1155/2022/7663659

**Published:** 2022-07-14

**Authors:** Man Wu

**Affiliations:** College of Art & Design, Nanjing Forestry University, Nanjing, Jiangsu, China

## Abstract

With the continuous development and progress of image sensing technology in recent years, the problem of image data acquisition, recovery, and recording has been solved, and people have gradually realized that image data can be better recovered, recorded, and exhibited by collecting image data. It is also used in target recognition, image display, landscape design, and other fields. And the application of color mapping algorithm can more intuitively affect the final quality of the display image. This is extremely important for landscape design. It can be said that the emergence and application of color mapping algorithm provide strong technical support for both dynamic and static image color automatic adjustment and simulation. On this basis, taking the color mapping algorithm as the breakthrough, through the in-depth introduction of the color mapping algorithm, starting from the direction of landscape image color automatic adjustment, a relatively simplified color mapping algorithm model inheriting the positive and negative two-way vision model is proposed. At the same time, a simulation algorithm based on landscape suitcase color automatic adjustment is proposed based on the color mapping algorithm model. Experiments show that automatic color adjustment of landscape images based on color mapping algorithm can achieve more realistic image reproduction, and the color mapping method based on color mapping algorithm has less illumination bias. When the number of experiments is 30, the difference in visibility of the plane is 0.25 cd/m^2^, the difference of visibility according to the color change segmented by the gradient area is 0.71 cd/m^2^, and the difference of the illuminance difference of the transition image is 0.71 cd/m^2^. Gaussian pyramid is 1.25 cd/m^2^. The proposed method improves color density by reducing image sharpness and compensating for color sharpness of landscape image, and high quality landscape images provide assistance for landscape design.

## 1. Introduction

Human visual perception is the most important way of human perception of the outside world. Due to the adaptability of human visual system (HVS) to the brightness of real-world scenes, we can perceive the illumination in a large dynamic range in real-world scenes. As an image processing system, the human visual system (HVS) is nonuniform and nonlinear in its perception of images. The visual characteristics of human eyes for images is mainly more sensitive to luminance signal than chrominance signal, sensitive to low-frequency signal than high-frequency signal, sensitive to still image than moving image, and sensitive to horizontal lines and vertical lines. In this way, we can not only see the dim stars at night, but also distinguish the color and details of objects in a sunny day. The scattering of natural light into the human eye makes HVS produces perceptual effect. Imaging technology seeks to use analog or digital array to simulate the scattered light reaching the human eye to provide us with an indirect “illusion” of perceiving the external real scene. Due to the development of modern colorology, people's understanding of color is increasing, which puts color in a very important position in people's life. Color is widely used in film and television, architecture, clothing, landscape design, and other fields. Color is a wonderful presentation, seen as a vision in everyday life. Information transmitted in color plays an irreplaceable role. From the expression of color, the symbolic function of color and the way of expression are explained. This paper emphasizes the transmission of color information and explains that the expression and symbol of color are used to convey different emotional information, making the picture fuller. How to obtain true color images through color matching is an important topic in various fields, and it is also an exception for landscape design. How to enhance the color and quality of landscape images is extremely important. This paper takes the color mapping algorithm as a breakthrough and proposes a relatively simplified color mapping algorithm model on the basis of inheriting the positive and negative two-way visual model. At the same time, based on the color mapping algorithm model, a simulation algorithm based on automatic color adjustment of landscape image is proposed for landscape design.

## 2. Literature Review

Zhang and others said that, in the past ten years, researchers have spent a lot of time and energy compressing the range of HDR images and videos to make the data visualization of LDR display more natural [1]. According to different processing methods, the existing algorithms are mainly divided into global algorithms and local algorithms. Ismail and others said that global mapping can maintain the overall effect of the image and make it easier to realize, but the algorithm using global image statistics cannot maintain the local contrast and the details of the original HDR image [2]. The local mapping adopts the comparison and calculation of pixels in a specific area, which can compensate the defects of the global mapping algorithm, but the operation speed is slow. Mohammadi and others said that the global algorithm based on *s* equation uses nonlinear function to compress the brightness range of the image, which can retain most of the detail information [3]. Some scholars have proposed an adaptive logarithmic mapping algorithm close to the logarithmic transformation characteristics of human eyes. The algorithm is fast, and the image color will not be distorted, but the limited compression range is easy to cause the loss of image details. Hidetoshi and others said that the layered algorithm assumes that, in the natural scene, the image is composed of slowly changing brightness information and jumping reflection components, and the more real natural information can be restored by dynamically compressing the brightness component and retaining the reflection component. The algorithm can obtain satisfactory results for the halo phenomenon and diffusion phenomenon [4]. Hu and others said that the tone mapping algorithm based on gradient domain regards the image as a two-dimensional discrete function. The original image is restored by constructing Gaussian pyramid and Poisson equation [5]. Yang and others said that, using the characteristics of human visual system and reducing image distortion by using high-order image data, the algorithm has a large amount of calculation [6]. Cai and others said that the probability model is used to realize the tone regeneration of the image, convert the tone mapping process into the problem of the maximum energy, and maintain the image visual information as much as possible [7]. Nong and others studied the algorithm of mapping the image by constructing piecewise linear function, extracted the image detail layer by bilateral filtering, and fused the brightness image and detail information to ensure the clear reproduction of the image texture [8]. Li and others said that the local multiscale Retinex mapping method is solved iteratively by regularization method, and the Retinex algorithm is used to eliminate the influence of illumination, so the image color fidelity effect is better. A fast detail-preserving algorithm is proposed, which has greatly improved the processing speed [9]. Liu and others said that the color correction method was used to solve the problem of color distortion in dynamic compression. The tone mapping algorithm based on photographic model uses the concepts of exposure and shading for different brightness to compress the dynamic range, which makes the algorithm more flexible. An algorithm based on multiscale Retinex is proposed, which realizes the compression of high dynamic range through the enhancement of brightness component, but it is easy to cause color distortion. Through the principal component analysis, the color space is transformed, and the guided filtering is used to realize the tone mapping. A tone mapping algorithm with controllable brightness and detail preservation is proposed. By estimating the image brightness and standard deviation, the brightness histogram is used for compensation, and the image detail contrast is improved [10]. The simulation of landscape image color automatic adjustment of color mapping algorithm is shown in Figure 1. In this paper, based on the previous research results, an image processing technology based on color mapping algorithm is proposed and applied to landscape image processing.

## 3. Method

Visible light is a type of radiant energy in the real world. The essence of light is electromagnetic waves. The sharpness value in an image with high dynamic range is a measure of the lighting information close to the surface of the object. It is a core parameter of tone mapping technology, and the frequency is usually 400–700 nm. In the process of propagation, natural light passes through the material, and the physical properties of the medium will change its propagation direction. Natural light has two physical properties: brightness and light radiation intensity. Brightness is the weight sum of spectral radiation intensity under various visible wavelengths. The calculation is shown in the following formula:

(1) $$\begin{array}{c} Y=\int_{380nm}^{780nm}L\left(\lambda \right)V\left(\lambda \right)\text{d}\lambda , \end{array}$$

where *V*(*λ*) is the spectral brightness efficiency curve. Some attributes of the scene can be described by the relative brightness of the scene. This relative measurement is called contrast. Contrast determines the relationship between the darkest and brightest values of these phenomena. Contrast refers to the measurement of different brightness levels between the brightest white and the darkest black in the light and dark areas of an image. The larger the difference range, the greater the contrast, and the smaller the difference range, the smaller the contrast. A good contrast ratio of 120 : 1 can easily display vivid and rich colors, and when the contrast ratio is as high as 300 : 1, it can support all levels of color. However, the contrast ratio suffers from the same dilemma as the brightness. There is no effective and fair standard to measure the contrast ratio, so the best way to identify it is to rely on the user's eyes. There are three commonly used comparisons: Weber comparison, Michelson comparison, and comparison. The definition is as follows:

(2) $$\begin{array}{c} C_{W}=\frac{L_{\max}-L_{\min}}{L_{\min}}, \end{array}$$

(3) $$\begin{array}{c} C_{M}=\frac{L_{\max}-L_{\min}}{L_{\max}+L_{\min}}, \end{array}$$

(4) $$\begin{array}{c} C_{R}=\frac{L_{\max}}{L_{\min}}. \end{array}$$

Our model is used for Weber contrast, Michelson contrast, and contrast difference. *L*_max_ and *L*_min_ represent the maximum illumination value and the minimum illumination value in the real scene. The neurological experiment uses an extremely simple natural image to measure visual adaptation. A short pulse light is superimposed on a uniform background. When the photoreceptor cells in the retina absorb the pulse intensity, the response curve of the photoreceptor cells of the cone and rod is calculated as shown in the following formula:

(5) $$\begin{array}{c} R=\frac{I^{n}}{I^{n}+I_{b}^{n}}. \end{array}$$

*I* is the intensity of light, *I*_*b*_ is the half-saturation constant, that is, the maximum intensity that can cause a human visual response, and *n* is the sensitivity control index. Color is the most vivid description of an image, so the research on color space is extremely important. The color consists of three primary colors. The three-dimensional mathematical description of color is called color space. The color space related to the device uses the same color to present different results on different display media, while the color information not related to the device does not depend on the specific media, and the output of the same color on different media is not different. The CIE 1931 XYZ color space is defined by the projection of the power distribution of the *I* spectrum onto a single color matching function. The calculation is as follows:

(6) $$\begin{array}{c} X=\int_{380}^{830}I\left(\lambda \right)\bar{x}\left(\lambda \right)\text{d}\lambda , \end{array}$$

(7) $$\begin{array}{c} Y=\int_{380}^{830}I\left(\lambda \right)\bar{y}\left(\lambda \right)\text{d}\lambda , \end{array}$$

(8) $$\begin{array}{c} X=\int_{380}^{830}I\left(\lambda \right)\bar{z}\left(\lambda \right)\text{d}\lambda . \end{array}$$

The chromaticity calculation of color is shown in the following formulae:

(9) $$\begin{array}{c} x=\frac{X}{X+Y+Z}, \end{array}$$

(10) $$\begin{array}{c} y=\frac{Y}{X+Y+Z}. \end{array}$$

The conversion calculation between RGB color space and XYZ color space is shown in the following formula:

(11) $$\begin{array}{c} \left[\begin{array}{c} X\\ Y\\ Z \end{array}\right]=M\left[\begin{array}{c} R\\ G\\ B \end{array}\right],\\ M=\left[\begin{array}{c} \begin{array}{ccc} 0.410 & 0.358 & 0.181 \end{array}\\ \begin{array}{ccc} 0.213 & 0.715 & 0.082 \end{array}\\ \begin{array}{ccc} 0.029 & 0.119 & 0.960 \end{array} \end{array}\right]. \end{array}$$

The physiological structure of HVS is extremely complex. Natural light intensity enters the human eye from the cornea, passes through the pupil, lens, retina, optic nerve, and other tissues, and then triggers visual perception in the visual cortex of the brain. Among them, the photoreceptors on the pupil and retina mainly affect the light intensity.

In fact, the change of pupil size is the response of background illumination brightness *L*_*a*_ [11]. In a specific environment, similar to the aperture in the camera, it can also be regarded as a protective device. In a bright environment, the contracted pupil can minimize the risk of retinal damage. In this case, the area size as of the pupil can be regarded as a function of the maximum adaptive brightness *L*_amax_, as shown in the following formula:

(12) $$\begin{array}{c} A_{s}=\pi {\left(2.45-1.5\;\tan\left(0.4\;\ln\left(L_{a\;\max}+1\right)\right)\right)}^{2}. \end{array}$$

The input natural light intensity can be converted to the light intensity on the retina by multiplying as, resulting in retinal brightness. Studies have shown that when HVS changes from bright sunlight to starlight at night. The diameter of pupil changes from about 2 mm to 8 mm. The properties of the human eye are largely determined by the structure of the human eye, including how light rays converge, how they are detected, and how visual signals are conducted. In addition, the characteristics of the nervous system, especially the human brain, also play a role in the processing of visual information. This change will only affect the natural light intensity of 16 times to enter the human eye. It can be seen from Table 1 that the variation range of natural light intensity is more than 100 million times. Therefore, the pupil is extremely limited to limit the entry of natural light into the human eye.

Photoreceptors on the retina are divided into rod cells and cone cells, as shown in Figure 2. Rod cells are extremely sensitive to light. From dusk to night, rod cells play a major role in human eyes. Cone cells are relatively less sensitive to light. This type of cells plays a role in the day to moonlight. Electrophysiological studies can be used to detect the response of individual nerve cells in HVS [12, 13]. The electrical response characteristics of a single cell are recorded by stimulating a thin electrode near or in the cell. The response characteristics correspond to the neural response of cone cells and rod cells to convert the light energy of the real scene into light energy. Compared with the large range of scene photography that the visual system can act on, the action range of the logarithmic curve response of the photoreceptor is extremely narrow, only three to four logarithmic units, as shown in Figure 2. The luminance response function curve in the log linear graph is obtained by measuring the electrical response of rod cells under different luminance values [14].

The shape of the response curve of cone cells is the same as that of rod cells. However, because the action range of rod cells and cone cells on light is different, the position of the response curve of cone cells is located on the right side of the logarithmic brightness axis. The light response curves of cone cells and rod cells are as shown in Figure 3.

The response curves of cone cells and rod cells can be expressed by Michaelis equation, as shown in the following formula:

(13) $$\begin{array}{c} R=\frac{I^{n}}{I^{n}+\sigma^{n}}. \end{array}$$

The initial saturation of photoreceptors occurs under illumination conditions about 100 times stronger than the background illumination, which is consistent with our empirical value of visual blinding brightness. However, this initial saturation value will not continue all the time. When the photoreceptor has been exposed to this light condition, the HVS will adapt to the environment, the saturation value will change, and the visual system can work normally again. Neurophysiological studies have shown that if photoreceptors are continuously exposed to high light conditions, the initial saturation value will not continue to be saturated, and the saturation value will move to the right after long-term exposure to high brightness conditions. Experiments under stable single light conditions show that the response curve is S-shaped. However, under gradually increasing light conditions, the position of the response curve will move parallel to the right along the *X*-axis. This movement shows that if there is sufficient time to adapt to the lighting conditions, the visual system always maintains the lighting response of three to four logarithmic units on the logarithmic brightness coordinate axis [15]. This movement can also be achieved by setting different *σ* value to complete the simulation, so rewrite formula (13) as the following formula:

(14) $$\begin{array}{c} R=\frac{I^{n}}{I^{n}+\sigma_{b}^{n}}. \end{array}$$

The above formula is the photoreceptor brightness adaptive model formula.

Converting the magnitude of physical change into the magnitude of perception is called Weber-Fechner law. Simply put, Weber-Fechner law gives that the magnitude of perceived stimulus is directly proportional to the logarithm of physical stimulus intensity [16, 17]. If Weber-Fechner law is strictly valid, then all perceptual relationships follow the same nonlinear form. Although the general trend of compression nonlinearity is suitable for most percepts, different percepts generally adopt functional relationships with different shapes, which means that Weber-Fechner law is not completely accurate. However, for the visual perception of human eyes, the results of many experiments obey Weber-Fechner law [18]. Because of its simplicity and efficiency, this law still has important reference significance for human visual perception modeling. Stevens used the numerical estimation method to study the relationship between 30 different types of perceptual physical stimuli and perceptual quantity. The results showed that the perceptual quantity curve was a straight line in the double log domain coordinate system, but the slope of the straight line corresponding to different perceptual types was different. Therefore, Stevens assumes that the relationship between perceptual quantity and stimulus intensity follows the power-law equation instead of Fechner's logarithmic equation. For human visual perception, the following formula is obtained:

(15) $$\begin{array}{c} s=I^{r}. \end{array}$$

Among them, *s* represents the visual value of the human eye to the natural world, *I* represents the light of the natural world, and *R* is the energy measurement unit determined by visible light and natural light. In order to obtain the value of power exponent *R*, Stevens used the numerical estimation method to obtain a large number of experimental data [19, 20]. The specific step is to present a standard light intensity stimulus to the tester and specify its occurrence value as a number, such as 1.00. Then, the tester takes this subjective value as the standard to judge other brightness stimuli with different intensities and expresses them with a number.  Table 2 shows the experimental results obtained.

The research of tone mapping based on visual physiology is based on the research results of human eye anatomy, neurophysiology, biochemistry, and biophysics to understand the structure and function of human visual organs, especially the formation mechanism of brightness compression of visual system under the condition of HDR natural scene, so as to construct a mathematical model and then carry out tone mapping operation on HDR image. The vision research based on psychology is to describe and analyze the relationship between brightness feeling, color feeling, and physical stimulation as much as possible, express how people “feel light” and “understand color” with mathematical model, and then apply the visual expression to HDR image to expect to get the same perception result on LDR display device. In order to further study this problem, we draw the mapping curves of the two visual perception models in the same coordinate system [21]. To make the algorithm more popular, we used low dynamic range light when displaying on low dynamic range display devices, and we assumed that the output range of accepted values is between 0 and 1. The photoreceptor sharpness response curve (solid line in the figure) is already in this range, as shown, but for the Weber-Fechner law curve (dotted line in the Figure), it must be normalized (midpoint line in the Figure 4).

The values of photoreceptor brightness response curve and Weber-Fechner law curve are extremely similar in the middle two orders (−1 to 1), but then, the photoreceptor brightness response curve will approach 1, and the Weber-Fechner law curve will continue to grow. This can be explained by the properties of photoreceptors: the cone curve only moves about 4 orders of magnitude. For higher brightness values, the cone will be saturated and lose sensitivity. Weber-Fechner law does not consider the saturation effect of cones, so the mapping curve will grow all the time. Light is reflected from the object surface into the human eye. If the HVS, like a camera, takes only one illumination measurement, it cannot differentiate between a white surface in the dark and a black surface in bright light. However, our eyes can distinguish these two situations well, which is called brightness constancy. The attributes of a typical natural scene include color, shadow, size, and shape, but these attributes are not clearly expressed in the retinal image, but through the processing of visual information transmission pathway. In order to extract these attributes, the luminance information must be spatially combined.

## 4. Experiment and Analysis

The testers participating in the subjective evaluation experiment should choose people with normal or normal vision and perform the relevant actions in strict accordance with the test steps. The tester collects information by interacting with the display interface. In order to avoid errors in the tester's judgment, an average gray image of the two images will be inserted when switching between one test image and the next test image [22].

The first is classification. First, HDR images were captured as LDR images through a multitone imaging algorithm, and each tester then classified the quality of this series of LDR images according to their choice. In this case, the evaluation results are more accurate because the tester has to determine the quality of each LDR image. The main disadvantage of this method is that the examiner has to compare all tests, which can take a long time to measure.

The second is the measurement method. The person evaluating the image quality will do so based on the measurement criteria. This method can be done quickly since there is no need for comparison with other pictures to try. However, this method is not that accurate because different experimenters give different measurements for the same image.

The real test of the map-guided algorithm is to study the similarity between the HVS image and the LDR image after the original HDR image, human perception. Therefore, this method is based on the simulation of HVS perception mechanism. Although the perception mechanism of HVS has been greatly developed in recent decades, there is no objective evaluation method of tone mapping in the world to completely simulate the perception mechanism of HVS, which only simulates some aspects of HVS. At present, HDR-VDP and DR are the most widely used objective evaluation methods of tone mapping. These two evaluation methods only aim at the brightness channel of the image and do not involve color information [23, 24].

HDR-VDP algorithm uses the contrast sensitivity function to filter the image, and then the algorithm decomposes the image into a series of subimages with different space and direction for differentiation calculation according to the response characteristics of human cerebral cortex to visual perception and visual mask. The phase uncertainty step is to remove the dependence of the phase on the mask [25]. Finally, the visual difference probabilities of all channels are added to produce a visual difference probability diagram, and the flow chart is shown in Figure 5.

The contrast detection step simulates the HVS mechanism, which is similar to HDR-VDP, and then uses the spatial transformation equation of cerebral cortex to model. The output contrast difference information is divided into different frequency bands through several band-pass filters with different filter core sizes and directions. Conditional probability is used to estimate the three contrast difference pieces of information in each frequency band. Finally, the three kinds of difference information are represented by different colors: green indicates the loss of visual perception of the contrast of the image to be tested; blue indicates that the visual perception of the contrast of the image to be tested is too strong; red indicates the visual perception reversal of the contrast of the image to be tested [26]. The flow chart of DRI algorithm is shown in Figure 6.

Since the objective evaluation method of DRI was proposed, it has been widely used to evaluate the advantages and disadvantages of tone mapping algorithm because of its excellent accuracy and ease of use. So far, many new authoritative tone mapping algorithms still take it as an objective evaluation standard. Although there are some objective evaluation methods for tone mapping later, the accuracy and applicability of evaluation need to be further verified. According to the image correction results given above, determine the response curves of channels *R*, *G*, and *B*, as shown in the following formula:

(16) $$\begin{array}{c} D\left(E\right)=\left(D_{\max}-D_{\min}\right)\times \frac{\log\left(E_{\min}\right)}{\log\left(E_{\max}\right)}. \end{array}$$

Among them, *E* represents the illuminance value of retro urban buildings, and *D* represents the gray value of retro urban buildings. *E*_max_ represents the maximum illuminance of urban retro buildings, and *E*_min_ represents the minimum illuminance of urban retro buildings. *D*_max_ represents the highest gray value of urban retro buildings, and *D*_min_ represents the minimum gray value of urban retro buildings. According to the above model, the average value of illuminance is shown in the following equation:

(17) $$\begin{array}{c} E_{\text{ave}}=\exp\left[\frac{1}{N}\sum_{x,y}\log+E\left(x,y\right)\right]. \end{array}$$

Here, *N* represents all pixels in the image, and *E*(*x*, *y*) represents the bright spot value. The median value is determined according to the following formula:

(18) $$\begin{array}{c} k=A\times B^{\left[2\;\log\;E_{\text{ave}}-\log\;E_{\max}\right]}. \end{array}$$

Among them, the value of *k* is [0, 1], and *A* and *B* represent constants. The offset of equation (18) is solved by the Newton iteration method, as shown in the following equation:

(19) $$\begin{array}{c} k=\frac{\log\left(E_{\text{ave}}+\tau \right)-\log\left(E_{\min}+\tau \right)}{\log\left(E_{\max}+\tau \right)-\log\left(E_{\min}+\tau \right)}, \end{array}$$

where *τ* is the offset. The color scale of the color channel is then mapped, and the color can be adjusted using a gain factor. It is necessary to model and verify the effect of the automatic color matching method of landscape image based on color mapping algorithm. The simulation environment is matlabr2015b, and the experimental data uses the otb-50 standard data set. The comparison results are shown in Table 3 [27, 28]. In Table 3, Et represents the number of experiments (Hours), Bd represents the color sharpness deviation (CD/m2), DM1 represents the landscape image color adjustment method based on the color mapping algorithm, Dm2 represents the gradient-based color adjustment method, and Dm3 represents a method for adjusting landscape images based on Gaussian pyramids.

As can be seen from Table 3, the color gamut difference according to the color painting algorithm is small. When the number of experiments is 30, the difference in visibility of the plane is 0.25 cd/m^2^, the difference of visibility according to the color change segmented by the gradient area is 0.71 cd/m^2^, and the difference of the illuminance difference of the transition landscape image is 0.71 cd/m^2^. Gaussian pyramid is 1.25 cd/m^2^. This program improves color fastness by reducing image sharpness and compensating for color sharpness. The color transition method based on color map algorithm and the color transition method based on gradient region segmentation are compared. Obviously, the landscape image color changing method according to the color chart has the advantage of the color changing method of dividing the medium color difference and the maximum color difference according to the gradation area. The color change method based on the minimum segmentation of the gradient area does not solve the color correction function, so. The picture is extremely different in color. By adjusting the color correction, this method can better reduce color distortion, maintain the pattern of the original image, and make the color combination better. Select a landscape image from the Otb-50 sample data set, and compare the color change time of the landscape image color change method according to the color mapping algorithm with the color change method according to the gradient area and the color change method according to the gradient area, segmentation. The comparison results are shown in Table 4. Dm stands for multiple methods, Dm1 stands for color shift based on graphics algorithm, Dm2 stands for color shift based on gradient region segmentation, and Dm3 stands for landscape image editing based on Gaussian pyramid, and the display time and display color change.

As shown in Table 4, the landscape image color change method based on the color mapping algorithm takes 1.23 seconds to adjust the color of the image. The color transition time of the color transition based on gradient region segmentation is 2.97 seconds. The set time for Gaussian pyramid-based landscape image correction is 3.63 seconds. This method has a shorter color change time than both methods. This method effectively reduces the color change time by adjusting the color of the landscape image.

## 5. Conclusion

Visual physiology studies have shown that the luminosity of the human eye is compressed into a large dynamic area in the real world, mainly by photoreceptors on the retina. Sound mapping algorithms based on photoreceptor sharpness adaptation models have been extensively studied. This paper analyzes the problems of existing algorithms and proposes an improved tone mapping algorithm. The new algorithm uses a local model based on the local features of the human eye space. The HDR image is first divided into three separate color channels, and then each color channel is routed and filtered to obtain the appropriate lighting value for each pixel of each color channel. Then, based on the photoreceptor brightness adaptive model, the characteristics of human photoreceptors with different response curves to different brightness levels of natural scenes are simulated. Finally, the color channels are combined to obtain the result landscape image. In this algorithm, an evaluation method for the key value *K* in the photoreceptor brightness adaptive model is also given, so that the algorithm does not need to set parameters manually, and the ease of use of the algorithm is improved. The algorithm simulates the brightness adaptive characteristics of human retinal photoreceptors, so it has a strong sense of reality. The adoption of local model makes the final landscape image have good visual visibility. Aiming at the defects of traditional methods, the gamma correction algorithm is used to correct the landscape image color, which effectively improves the landscape image color recognition rate and provides a certain guarantee for further color adjustment. The color mapping adjustment algorithm is used to adjust the color of the landscape image, which reduces the color brightness deviation in the process of image recognition, minimizes the color difference, and effectively improves the effect of color adjustment. This method is extremely effective in improving the quality of landscape image and can be used in landscape design, but it needs to be further improved. How to automatically match with landscape design and realize the integration of landscape design and landscape image processing is the focus of the next stage of research.

## Figures and Tables

**Figure 1:** Simulation of automatic color adjustment of landscape image based on color mapping algorithm.

**Figure 2:** Response of rod cells to dark adaptation under different brightness values.

**Figure 3:** Response curves of rod cells and cone cells under various light intensities.

**Figure 4:** Compares the response curves of different perception types.

**Figure 5:** Flow chart of HDR-VDP algorithm.

**Figure 6:** RI algorithm flow chart.

**Table 1:** Brightness values of typical natural scenes.

Natural scene	Brightness value (cd/m^2^)
Night sky	0.001
Waning moon	0.01
Full moon	0.1
Evening	1
Overcast	100
Sunny day	10000
Scorching sun	100000

**Table 2:** Stevens numerical estimation.

Light intensity	1	2	3	4	5	6	7	8	9	10

Psychological quantity	1	1.24	1.42	1.58	1.70	1.81	1.90	2.00	2.06	2.14

**Table 3:** Comparison of landscape image brightness deviation of different methods.

Et/(times)	Dm1	Dm2	Dm3
10	0.24	0.58	0.62
20	0.27	0.69	0.86
30	0.25	0.71	1.25

**Table 4:** Comparison of color adjustment time of different methods.

Dm	Time (s)
Dm1	1.23
Dm2	2.97
Dm3	3.63

## Data Availability

The data used to support the findings of this study are available from the corresponding author upon request.
